# The Anti-inflammatory Effect of Chitosan Oligosaccharide on Heart Failure in Mice

This article has been retracted.

**DOI:** 10.1155/2022/8746530

**Published:** 2022-10-05

**Authors:** Yubiao Zhang, Yu Wang, Yunen Liu, Tianxing Gong, Mingxiao Hou

**Affiliations:** ^1^Department of Food Science, Shenyang Agricultural University, No. 120 Dongling Road, Shenhe District, Shenyang, Liaoning, China 110866; ^2^Emergency Medicine Department of General Hospital of Northern Theater Command, Laboratory of Rescue Center of Severe Wound and Trauma PLA, No. 83 Wenhua Road, Shenhe District, Shenyang, Liaoning, China 110016; ^3^Sino-Dutch Biomedical and Information Engineering School, Northeastern University, No. 195 Chuangxin Road, Hunnan District, Shenyang, Liaoning, China 110169

## Abstract

Heart failure is currently one of the leading causes of death worldwide, and the inflammatory factors play an important role in its development. Chitosan oligosaccharide (COS), a low-molecular-weight form of chitosan, has many specific biological activities. In this study, COS effects on heart failure were studied for the first time by performing transverse arch constriction (TAC) surgery in mice, as an animal model of heart failure. Our findings revealed that COS administration (in both 40 mg/kg and 80 mg/kg doses) significantly ameliorated TCA-induced left ventricular (LV) hypertrophy as well as the increase in lung and heart weight in mice, while improving TAC-induced LV dysfunction. Both doses effectively attenuated LV cardiomyocyte hypertrophy, while decreasing heart inflammation after heart failure in mice. In conclusion, our results indicated that the supplementation of COS in normal diet might be an effective way to prevent further myocardial tissue damage in patients suffering from heart failure.

## 1. Introduction

Hear failure is the end-stage manifestation of cardiac dysfunction, indicating that the heart can no longer serve as a pump supporting physiological circulation [1–3]. Heart failure can be caused by ischemic heart disease, myocarditis, cardiomyopathy, and myocardial infarction. Heart failure is becoming a significant global concern. When these cardiovascular diseases occur, the myocardial contractile function will gradually decline; end-stage heart failure will eventually follow after the hemodynamic disorder is intensified [3–5]. In addition, heart disease is recognized as the leading cause of death in the worldwide. According to the American Heart Association, about 6 million patients are admitted for treatment due to heart failure in the U.S. each year [6, 7].

Chitosan is the only pseudonatural cationic polymer comprised of glucosamine (*β* (1-4)-linked 2-amino-2-deoxy-D-glucose) and N-acetylglucosamine (2-acetamido-2-deoxy-D-glucose) and is usually prepared by deacetylation of chitin. Chitin primarily found in exoskeletons of insects and crustaceans and is the second most abundant naturally occurring polymer after cellulose [7, 8]. Chitosan is following the protonation of primary amino groups of glucosamine in the C2 position and is mildly toxic, nonimmunogenic, biodegradable, and soluble in acidic aqueous solutions. As a result, it has been widely studied and is extensively used for biomedical and pharmaceutical applications [9–11].

Chitosan oligosaccharide (COS) is a low-molecular-weight form of chitosan, but it is soluble in neural pH solutions due to its short chain length. Therefore, it has many beneficial biological functions, including antifungal, antibacterial, antitumor, anti-infection, and immunity enhancing [12, 13]. Furthermore, COS can be easily absorbed through intestinal epithelium and quickly enters systemic circulation. It is shown that COS can enhance the phagocytic activity of macrophages by a mechanism related to nicotinamide adenine dinucleotide phosphate (NADPH) oxidase, which induces nitric oxide synthase (i-NOS) [14–16]. Several studies have demonstrated protective effects of COS on damaged cardiomyocytes. For example, available evidence is indicated that COS improves the antioxidant capacity of myocardial tissue during vigorous exercise, helps maintain the normal morphological structure of cardiac tissue, and prevents heavy-load exercise-induced myocardial damage [17, 18]. COS can reduce the mortality of LPS-induced sepsis mouse model, inhibit the inflammatory reaction in the whole province, and reduce the TNF in the serum-*α* and IL-1 content to reduce the damage to the liver, kidney, and lung [13]. However, to the best of our knowledge, the protective effects of COS on heart failure have not been previously investigated.

COS was fed to male mice for two weeks, and heart failure was subsequently induced to evaluate the protective effects of COS on heart failure progression. The expressions of inflammatory-specific genes and proteins were characterized to investigate the mechanisms of protective effects of COS on heart failure.

## 2. Material and Methods

### 2.1. Material

COS (Mn 1,000 Da, >90% deacetylation degree) was prepared by the enzymatic method at the Dalian Institute of Chemical Physics and was kindly provided for this investigation. COS was analyzed by Time-of-Flight Mass Spectrometry (TOF-MS, Agilent, U.S.A.).

### 2.2. Animal Model

The animal study was approved by the animal welfare committee of Shenyang Military Command Hospital (Permit No. 2020-014).

The animal studies conducted as a part of this investigation were approved by the Animal Care and Use Committee of the Northern Theater General Hospital. The study sample included forty 8- to 10-week-old male BALB/c mice obtained from Liaoning Provincial Laboratory Animal Public Service Center. The Laboratory Animal Public Service Center of Liaoning Province provides free food and water for small animals. After one-week acclimation, the animals were randomly divided into four groups (*n* = 10), namely, the sham operation group (control), the group in which the transverse arch constriction (TAC) surgery was performed to induce heart failure and mice were fed normal diet (the TAC group), the two intervention groups, in which the TAC surgery was also performed but mice were fed COS-supplemented (40 mg/kg or 80 mg/kg) diet every day for two weeks prior to surgery, denoted as the TAC-40COS and TAC-80COS groups, respectively.

The purpose of TAC surgery was to induce heart failure. In brief, mice were anesthetized by the intraperitoneal injection of sodium pentobarbital (50 mg/kg, Sigma, U.S.A.), and surgery was performed by an experienced surgeon. Subsequently, the aorta was ligated between the right and left common carotid arteries with a 27-gauge needle and 8-0 sutures. After surgery, mice assigned to the TAC-40COS and TAC-80COS groups were continuously fed with COS-supplemented food for additional four weeks, while those assigned to the control and the TAC group were provided normal diet. At the endpoint (after four weeks postsurgery), mice were euthanized by pentobarbital sodium injection (50 mg/kg).

### 2.3. Echocardiographic Assessment

Prior to euthanization, mice were anesthetized and evaluated for cardiac geometry and function by animal echocardiography (Vevo 770, Fujifilm, Japan). The anterior and posterior wall dimensions of the left ventricle (LV) were determined from three consecutive cycles during one cycle of diastole and systole. Fractional shortening was defined as the ratio of the duration from LV end-diastolic to end-systolic diameters.

### 2.4. Tissue and Plasma Collection

Blood samples were collected in anticlotting tubes from abdominal arteries and centrifuged at 7500 rpm for 15 min. Only the top layer of plasma was collected and was stored at -80°C for future use. In addition, cardiac tissues were collected with cryovials and were immediately preserved at -80°C.

### 2.5. Histological Analysis

Tissues were fixed in 10% formaldehyde solution for more than 72 h and then dehydrated and embedded in paraffin. Slices of 5 *μ*m thickness were prepared by a microsystem microtome (Leica RM2265, Germany) and were stained with hematoxylin-eosin (H&E, Sigma-Aldrich, U.S.A.) and Masson trichrome (Sigma-Aldrich, U.S.A.). Subsequently, stained slices were observed under light microscope (BX53, Olympus, Japan) to investigate cellular morphology and fibrosis.

### 2.6. Biomarker Analysis

In the present study, malondialdehyde (MDA) and superoxide dismutase (SOD) from serum were evaluated by the enzyme-linked immunosorbent assay (ELISA) method. The ELISA kit was purchased from IBL Company (Germany). In brief, the plasma samples stored at -80°C were thawed at room temperature, and 10 *μ*L drops of plasma were transferred to the 96-well plate provided in the ELISA kit. The reagents included in the kit were added into each well according to the manufacturer's instructions. The plate was incubated at 37°C for 10 min away from light and was subsequently read in the microplate reader (CLARIOstar, BMG, Germany) at the wavelength of 450 nm (*n* = 10 biological replicates).

### 2.7. Genetic Analysis

The genes related to the development of inflammation (IL-1*β*, IL-6, TNF-*α*, IL-17, NF-*κ*B, TGF-*β*, and smad1) were evaluated in this study, and the *β*-actin gene was used as the housekeeping gene. Using the RNeasy Mini Kit (Qiagen, Texas, U.S.A.), total RNA was isolated from the stored tissue samples and was reversely transcribed to cDNA on the thermal cycler (Bio-Rad, U.S.A.). Subsequently, the cDNA mixtures were amplified via real-time PCR (CFX96, Bio-Rad, U.S.A.) which involved the following steps: initialization at 95°C for 10 min, denaturation at 95°C for 15 s, annealing at 55°C, and extension at 68°C, repeated for 40 cycles. In the data analysis, the fold changes of each gene were calculated by applying the 2^-*ΔΔ*Ct^ formula, and the relative fold change was calculated as the fold change sample/fold change control ratio based on 10 biological replicates.

### 2.8. Western Blot Analysis

In this study, the Western blot method was adopted to analyze the expressions of proteins related of inflammation. In brief, tissue samples were homogenized (TissueLyser II, Qiagen, U.S.A.), and 160 *μ*L of tissue homogenate was separated in the electrophoresis chamber (Mini-PROTEAN, Bio-Rad, U.S.A.) on the SDS-PAGE gels (Mini-PROTEAN TGX gel, Bio-Rad, U.S.A.). Subsequently, the gels were transferred onto the PVDF membranes (Immun-Blot, Bio-Rad, U.S.A.) in the Western blotting transfer system (Trans-Blot Turbo, Bio-Rad, U.S.A.). The membranes were then incubated with the primary antibodies (rabbit anti-mouse, Abcam, U.S.A.) overnight and were washed with cold PBS to rinse antibody residue before further 4-hour incubation with the secondary antibodies (goat anti-rabbit, Abcam, U.S.A.). Finally, the antibody-bound membranes were observed in the imaging system (ChemiDoc MP system, Bio-Rad, U.S.A.) to analyze the protein expressions.

### 2.9. Statistical Analysis

The SPSS software (version 19.0, U.S.A.) was used for all statistical analyses, and one-way ANOVA was performed to determine the significance of between-group differences (*p* < 0.05).

## 3. Results and Discussion

As shown in Figure 1, the weight of left ventricle (Figure 1(a)), left atrium (Figure 1(b)), whole heart (Figure 1(c)), and lung (Figure 1(d)); the ratio of left ventricle (LV) weight to tibial length (Figure 1(e)); and the ratio of left atrium (LA) weight to tibial length (Figure 1(f)) of the TAC surgery significantly increased. Moreover, the mice were fed COS-supplemented diet; hypertrophy of aforementioned tissues was significantly reduced, indicating that COS might have some protective effects against heart failure. Furthermore, as can be seen from Figure 1, the tissue weights were lower in the TAC-80COS relative to the TAC-40COS group. Although the difference was not statistically significant, these findings suggest that the protective effects of COS might be concentration-dependent. Heart failure leads to elevated inflammatory cytokines, which in turn causes inhibition of myocardial contraction and subsequent hypertrophy and apoptosis of cardiomyocyte [19–21]. These findings are in line with the results reported by Hanna and Frangogiannis and Zhou and Qian, who noted that gavage of COS to pollution-affected rats significantly reduced the extent of lung injury in a dose-dependent manner [22, 23]. These effects may be attributed to the ability of COS to counteract the oxidative stress induced by the TAC surgery.

The ultrasound heart function assessments are depicted in Figure 2. As can be seen from Figures 2(a) and 2(b), both the end-diastolic and end-systolic diameters in the left ventricle (LV) increased as a result of heart failure induced by TAC surgery and decreased due to administration of COS. Moreover, the ejection fraction (LVEF) and the ejection fractional shortening (LVFS) of the left ventricle, depicted in Figures 2(c) and 2(d), respectively, were significantly reduced as a result of heart failure and improved due to COS supplementation. Furthermore, as shown in Figures 2(e) and 2(f), the minimum and the maximum increase and decrease rates in LV were also affected by heart failure and improved due to COS. In this present work, we evaluated the cardiac functions in LV. The changes in these functions strongly indicate that heart failure was successfully induced in mice by the TAC surgery. The results presented in Figures 1 and 2 confirm that COS has effect on cardiac tissue protection from heart failure but warranted further analyses to investigate the protective mechanism of COS in heart failure.

The H&E and Masson staining results are presented in Figures 3 and 4, respectively, to examine the pathological changes of cardiomyocytes. As can be seen in Figure 3(a), the nuclei of cardiomyocytes were purple/blue, and the cytoplasm was gray, confirming that cardiomyocytes were normal in the control group. In the TAC group (Figure 3(b)), hypertrophy was observed, along with cardiomyocytes, accompanied by the infiltrated inflammatory cells. In Figures 3(c) and 3(d), pertaining to the two groups that were fed COS-supplemented diet, hypertrophy could also be noted along with cardiomyocytes, while the number of inflammatory cells was lower than in the TAC group. Similarly, Figure 4 shows that no fibrosis was present in cardiac tissues in the control group (Figure 4(a)), while serious tissue fibrosis was observed in the TAC group (Figure 4(b)). In addition, six-week COS supplementation significantly reduced myocardial fibrosis (Figures 4(c) and 4(d)). These results strongly indicate that COS could reduce cardiac hypertrophy and the infiltration of inflammatory cells resulting from heart failure.

The MDA and SOD were investigated to evaluate and compare the oxidative stress levels in mice that suffered heart failure (the TAC, TAC-40COS, and TAC-80COS groups). As shown in Figure 5(a), the MDA level in the control group (Figure 5(a)) was significantly lower than in the other three groups. On the other hand, the SOD level (Figure 5(b)) in the control group was significantly higher than in the other three groups. Because both biomarkers are closely related to oxidative stress, the elevation of MDA and reduction in SOD strongly indicate that myocardial tissues were severely affected by heart failure. In addition, these results are consistent with the findings yielded by the aforementioned analyses, suggesting that COS supplementation plays a protective role against heart failure.

IL-17 is an early T cell-induced inflammatory response initiator, which can amplify the inflammatory response by promoting the release of proinflammatory cytokines. IL-17 plays its biological role through the MAP kinase pathway and nuclear factor KB (NF-*κ*B) pathway after binding to receptors [24–26]. The inflammation-specific gene and protein expressions are shown in Figures 6 and 7, respectively. Cytokine nf-*κ*b, encoded by nf-*κ*b gene, is an inflammatory factor and controls the nuclear transcription factor. Cytokine IL-17 induces nf-*κ*b activation, which in turn promotes the expressions of IL-1*β*, IL-6, and TNF-*α*, thereby accelerating the inflammatory response in heart tissues and leading to cardiomyocyte apoptosis, eventually lead to heart failure. Our results indicate that both genetic and protein expressions of the aforementioned factors significantly increased as a result of TAC surgery but were reduced by COS supplementation (*p* < 0.05). As a signal pathway downstream of MyD88, NF-*κ*B p65 is a key transcription factor in the inflammatory response, NF-*κ*B in resting state with inactive I *κ* B/NF-*κ*B form of complex exists in the cytoplasm. NF-*κ*B can promote gene transcription of cytokines, chemokines, and inflammatory factors and amplify inflammatory signals after activation [27, 28]. TGF-*β* promotes inflammatory response and accelerates heart failure development with the downstream effector of smad1. Our analyses indicate that both TGF-*β* and smad1 expressions were significantly upregulated by the TAC surgery (Figure 7) as compared to the control group (*p* < 0.05) and were reduced by COS supplementation. These gene analysis results are confirmed by Western blot images shown in Figure 7. TGF-*β* makes inflammatory macrophages ineffective and promotes myofibroblast transdifferentiation and matrix synthesis through the Smad protein-dependent pathway. Smad1 also plays a certain role in the process of inflammation [29]. Moreover, the statistically significant differences between the findings obtained for the TAC-40COS and TAC-80COS groups indicate that the role of COS in heart failure prevention is concentration-dependent. Based upon the above analysis, it can be surmised that COS could protect myocardial tissues from heart failure by suppressing the expression of inflammation-specific factors in a concentration-dependent manner.

## 4. Conclusion

In conclusion, as a part of this investigation, we induced heart failure in mice by performing TAC surgery and supplemented two groups with different doses of COS to assess its protective effects against heart failure. Our results reveal that COS supplementation could significantly suppress the expressions of inflammation-specific factors, such as TNF-*α*, and can thus protect myocardial tissues from further damage. These findings indicate that COS should be considered as a functional dietary supplement for patients that have suffered cardiac damage in order to prevent further exacerbation of their condition. Therefore, further studies are needed to comprehensively evaluate COS biosafety in these future applications.

## Figures and Tables

**Figure 1:** COS scavenger attenuates ventricular hypertrophy and pulmonary congestion in response to systolic overload. (a) The ratio of left ventricle (LV) to body weight of mice. (b) The ratio of left atrium (LA) to body weight of mice. (c) The ratio of heart to body weight of mice. (d) The ratio of lung to body weight of mice. (e) The ratio of left ventricle (LV) weight to tibial length. (f) The ratio of left atrium (LA) weight to tibial length. ^∗^*p* < 0.05, compared to the sham group, and #*p* < 0.05, compared to TAC group. All values are mean ± SEM.

**Figure 2:** Echocardiographic and hemodynamic measurements demonstrating that COS scavenger attenuate TAC-induced left ventricular hypertrophy and dysfunction. (a, b) Summary data from echocardiograms measurements of LV end-diastolic diameter and LV end-systolic diameter. (c, d) Summary data from echocardiogram measurements of LV ejection fraction and LV fraction shortening. (e, f) LV maximum rate of rise of pressure (dP/dtmax) and LV maximum rate of decline of pressure (dP/dtmin) from hearts. ^∗^*p* < 0.05, compared to the sham group, and #*p* < 0.05, compared to the TAC group. All values are mean ± SEM.

**Figure 3:** HE staining of heart: (a) Sham group; (b) TAC group; (c) TAC+40 mg/kg COS group; (d) TAC+80 mg/kg COS group.

**Figure 4:** COS attenuated TAC heart fibrosis: (a) sham group; (b) TAC group; (c) TAC+40 mg/kg COS group; (d) TAC+80 mg/kg COS group.

**Figure 5:** Changes of myocardial antioxidant enzymes under cold exposure. (a) The content of MDA in mouse serum. (b) The content of SOD in mouse serum. ^∗^*p* < 0.05, compared to the sham group, and #*p* < 0.05, compared to the TAC group. All values are mean ± SEM.

**Figure 6:** Inflammatory proteins and gene in myocardium under TAC. (a) Western blotting images of IL-1*β*, IL-6, IL-17, TNF-*α*, and nf-*κ*b in four groups. (b) The gene expression of IL-1*β*. (c) The gene expression of IL-6. (d) Gene expression of il-17. (e) The gene expression of TNF-*α*. (f) The gene expression of nf-*κ*b. ^∗^*p* < 0.05, compared to the sham group, and #*p* < 0.05, compared to TAC group. All values are mean ± SEM.

**Figure 7:** Inflammatory proteins and gene in TGF-*β*/smad1 signal pathway. (a) Western blotting images of TGF-*β* and smad1 in four groups. (b) The gene expression of smad1. (c) The gene expression of TGF-*β*. ^∗^*p* < 0.05, compared to the sham group, and #*p* < 0.05, compared to the TAC group. All values are mean ± SEM.

## Data Availability

The datasets used and/or analyzed during the current study are available from the corresponding author on reasonable request.
